# Language aptitude in the visuospatial modality: L2 British Sign Language acquisition and cognitive skills in British Sign Language-English interpreting students

**DOI:** 10.3389/fpsyg.2022.932370

**Published:** 2022-09-14

**Authors:** Freya Watkins, Stacey Webb, Christopher Stone, Robin L. Thompson

**Affiliations:** ^1^Multimodal Multilingual Language Processing Lab, School of Psychology, University of Birmingham, Birmingham, United Kingdom; ^2^School of Social Sciences, Languages and Intercultural Studies, Heriot-Watt University, Edinburgh, United Kingdom; ^3^School of Social, Historical and Political Studies, University of Wolverhampton, Wolverhampton, United Kingdom

**Keywords:** sign language, interpreting, cognition, language aptitude, L2 acquisition

## Abstract

Sign language interpreting (SLI) is a cognitively challenging task performed mostly by second language learners (i.e., not raised using a sign language as a home language). SLI students must first gain language fluency in a new visuospatial modality and then move between spoken and signed modalities as they interpret. As a result, many students plateau before reaching working fluency, and SLI training program drop-out rates are high. However, we know little about the requisite skills to become a successful interpreter: the few existing studies investigating SLI aptitude in terms of linguistic and cognitive skills lack baseline measures. Here we report a 3-year exploratory longitudinal skills assessments study with British Sign Language (BSL)-English SLI students at two universities (*n* = 33). Our aims were two-fold: first, to better understand the prerequisite skills that lead to successful SLI outcomes; second, to better understand how signing and interpreting skills impact other aspects of cognition. A battery of tasks was completed at four time points to assess skills, including but not limited to: multimodal and unimodal working memory, 2-dimensional and 3-dimensional mental rotation (MR), and English comprehension. Dependent measures were BSL and SLI course grades, BSL reproduction tests, and consecutive SLI tasks. Results reveal that initial BSL proficiency and 2D-MR were associated with selection for the degree program, while visuospatial working memory was linked to continuing with the program. 3D-MR improved throughout the degree, alongside some limited gains in auditory, visuospatial, and multimodal working memory tasks. Visuospatial working memory and MR were the skills closest associated with BSL and SLI outcomes, particularly those tasks involving sign language production, thus, highlighting the importance of cognition related to the visuospatial modality. These preliminary data will inform SLI training programs, from applicant selection to curriculum design.

## Introduction

### Background and situation of sign language interpreting training in universities

Sign language interpreting (SLI) is known to be a uniquely challenging task, but few studies have investigated the linguistic and cognitive skills that make a prospective student interpreter more likely to succeed. In Great Britain, one of the main routes to becoming a sign language interpreter is completing a 3- to 4-year SLI undergraduate degree, where students acquire the target sign language (British Sign Language; BSL) alongside developing their interpreting skills. Both sign language learning and learning to interpret are challenging and distinct endeavors and likely due to these challenges, SLI degree programs suffer from high drop-out rates (see e.g., Grbić, 2009; Leitner, 2012; Huhtinen, 2014). First, unlike spoken language interpretation, where many interpreters are bilingual in both their working languages from an early age, the majority of SLI students do not enter programs with pre-existing sign language fluency and, thus, their initial second language (L2) acquisition occurs within a university, and not community, context (Cokely, 1986; Peterson, 1999; Monikowski and Peterson, 2005). Furthermore, there may be special challenges involved in learning an L2 in a different modality. Concerningly, there is evidence that the academic demands of SLI degrees mean that students have fewer opportunities to engage with the deaf community (Pivac, 2014); that SLI students overestimate their sign language fluency and interpreting skills (Beal et al., 2018; Robinson and Henner, 2018); and that many do not attain working sign language fluency even by the end of their degree programs (see e.g., Volk, 2014). Together, these contribute to a gap between SLI training completion and competent practice (Witter-Merithew and Johnson, 2005).

As well as learning an L2 in a new modality during their degree program, SLI students also must learn how to interpret. SLI is both cognitively and linguistically demanding, involving the simultaneous use of two languages in two different modalities (Padden, 2000). However, there is minimal research into whether a cognitive aptitude profile exists for L2 SLI students embarking on the study to reach professional fluency. Here, we follow López Gómez et al. (2007), who found that perceptual-motor skills and cognitive verbal abilities played a greater role than personality in predicting SLI students’ sign language proficiency, suggesting that greater focus should be placed on cognitive predictors of signing and interpreting outcomes, as does Stone (2017). While a lot of research on cognitive aptitude for spoken interpreters exists, some of this is modality-specific and only applicable to the spoken-language aspects of SLI. It is also less informative regarding the cognitive and linguistic skills required to interpret sign language in the visuospatial modality. Another important difference is that spoken language interpreters work primarily from their L2 into their L1, whereas most signed language interpreters work primarily from spoken L1 into signed L2 (Nicodemus and Emmorey, 2013). Assessing linguistic and cognitive aptitude for SLI prior to entry into interpreter training programs could help reduce drop-out rates, minimize the rehousing of struggling SLI degree students into Deaf Studies programs (Stone, 2017), and would ultimately save a lot of time, both for instructors and students. According to Grbić (2009), beginner SLI students are often motivated by “social goodwill” but are less aware of the cognitive, social, and emotional demands of SLI, which initial pre-screening may help to highlight. Assessment at intake is, thus, not aimed at discouraging L2 sign language learning or potential SLI students, but, instead, encourages them to recognize as early as possible that SLI is challenging for various reasons.

Importantly, incomplete L2 sign language acquisition or insufficient skill in interpreting results in a lack of language access for deaf people who may use SLI services and when interacting with hearing people who do not sign. In the United Kingdom (UK), demand for SLI services frequently exceeds supply (Department for Work and Pensions [DWP], 2017). This can, in turn, lead to the use of unqualified, non-professional language brokers who do not meet the national standards for interpreting (CFA, 2012). Understanding the linguistic and cognitive factors that are important for both successful L2 sign language acquisition and high-level interpreting, is, thus key to improving access for deaf people.

Furthermore, training SLI students involves a significant financial investment. Whether students self-funded their studies or are supported by government grants, it is vital to ensure that the limited resources in SLI training (Webb, 2017) are used sensibly, and those students with optimum potential are supported. As Hunt and Nicodemus (2014) point out: “[o]ne of the problems with gatekeeping is timing; by the time a student gives evidence that they are not suitable, they have already invested a great deal of time and money in their degree.” While aptitude testing on admission is considered integral and is a standard practice in spoken language interpreting courses (see, e.g., Timarová and Ungoed-Thomas, 2008), SLI degree programs in the UK do not presently use any research-informed methods to test applicants in terms of their suitability (Stone, 2017). In the United States, the assessment of cognitive skills was found to be only a minor aspect of SLI programs’ entrance requirements (Marks, 2014), with most institutions focusing only on American Sign Language (ASL) and English skills. In Australia, initial SLI degree screening has been found to be informal and is often not evidence-based (Bontempo and Napier, 2009). Initial data highlighting which cognitive and linguistic assessments are likely related to SLI aptitude would therefore also be a benefit to prospective students and SLI programs.

### Cognitive and linguistic skills in spoken language interpreting

In spoken language interpreting, it has long been known that cognitive skills like working memory and cognitive load are vital to the interpreting process (see, e.g., Gile, 1997) and thus an important consideration for interpreter educators. As a result, cognitive aptitude for spoken language interpreting has been investigated to a greater extent than for SLI, with research now spanning several decades (for review, see Russo, 2011). This means that some aptitude test batteries have been validated for their reliability and are now widely used to screen spoken language interpreting trainee candidates or for intensive language training programs. For example, many interpreter training programs use long-standing commercial aptitude batteries like the Modern Language Aptitude Test (MLAT, Carroll and Sapon, 1959; Carroll et al., 2010) or the Pimsleur Language Aptitude Battery (Pimsleur, 1966), which include tasks involving learning new vocabulary and phonetic discrimination, among others.

More recently, research has focused particularly on the importance of working memory (WM) in spoken language interpreting, however, the findings are mixed. Both improvements in WM after interpreting training (Christoffels et al., 2006; Babcock et al., 2017; Chmiel, 2018) and WM effects on simultaneous interpreting fluency (Lin et al., 2018) have been reported. Auditory WM has also been shown to be more important than social factors like personality in simultaneous spoken language interpreting (Anssari-Naim, 2021), and L2 auditory WM is correlated with consecutive interpreting performance (Dong et al., 2018). However, some studies found no effects of WM: for example, professional interpreters were no different in general WM capacity from beginner interpreter students (Liu et al., 2004); linguistic factors, such as word knowledge in L1 and L2, were more important for interpreting performance than increased WM capacity (e.g., Padilla et al., 2005), and interpreting training has been found to improve language processing skills, but not WM (Tzou et al., 2012). In terms of other cognitive skills, spoken language interpreters have been shown to have superior cognitive flexibility over bilinguals with no interpreting training (Yudes et al., 2011), as well as superior dual-task attention compared to non-interpreters (Morales et al., 2015; Strobach et al., 2015). Macnamara (2009) also provides a review of cognitive functions and capacities required for interpreting, including chunking, online decision-making, and processing speed.

In this preliminary study, we focus on sign language interpreters who, like spoken language interpreters, make use of auditory WM, but also need to rely on visuospatial WM. According to Baddeley’s model of WM (Baddeley et al., 2009; Baddeley, 2012), auditory memory and visual memory are maintained through separate functional components: the phonological loop, and the visual sketchpad, respectively. This suggests that there may be different memory requirements or processes for SLI compared to spoken language interpreting, given the different modalities that must be attended to.

### Existing work on linguistic and cognitive aptitude for sign language interpreting

As with spoken language interpreting, there has been a long-standing interest in establishing which skills are required to be successful in SLI (for review, see Nakano, 2021). Some studies have taken the approach of surveying and studying the attributes of qualified sign language interpreters (e.g., Jones and Quigley, 1974; Seal, 2004; Shaw and Hughes, 2006), the latter finding that visual attention while inhibiting distractors was a particularly important skill. Other studies have compared skills in signed and spoken language interpretating students. For example, Shaw (2011) found better visual memory skills and concentration in SLI students than in spoken language interpreting students, both in terms of longer retention of visual information and better performance when visual distractors were present. Other linguistic and cognitive aptitudes that have been mentioned in the literature for both spoken language interpreting and SLI include a high command of both working languages, verbal fluency, processing speed, good WM, and concentration. For SLI alone, a further factor was the capacity to sign and talk simultaneously (Frishberg, 1986; Lara Burgos and de los Santos Rodríguez, 2000; cited in López Gómez et al., 2007).

Researchers have also explored the role of WM in SLI, again with mixed results. Wang (2016) found no evidence that auditory WM capacity in English or visual WM in Auslan was related to SLI task performance in either direction. However, van Dijk et al. (2012) found that auditory WM span in Dutch and visual WM in Sign Language of the Netherlands (NGT) were related to the quality of interpretations by NGT-Dutch interpreters. Looking at domain-general cognitive skills beyond WM, Macnamara et al. (2011) found that highly-skilled ASL-English interpreters had greater mental flexibility, faster cognitive processing, and psychomotor speed, and were better at task-switching when compared to less-skilled interpreters. Haug et al. (2019a,b) described initial data from working Swiss German Sign Language (DSGS)-German interpreters on a battery of cognitive tasks, developing their versions of WM tasks featuring DSGS stimuli. Their preliminary results suggest that the cognitive abilities of interpreters on all normed tests are above average, and that weaknesses or average performance in certain cognitive areas may be compensated by strengths in others. Studies on cognition in qualified working interpreters can inform us about the ‘end results’ of SLI training and professional experience, but are less informative regarding prospective SLI students: it is not clear which skills were improved through SLI training or professional experience, or if some skills are foundational and should ideally be at a threshold level at the outset of learning.

In terms of students, some SLI educators have administered broad pre-admission test batteries before SLI training, finding predictive relationships between performance in the screening battery and later SLI outcomes (e.g., Humphrey, 1994; Bontempo and Napier, 2009). However, only the cumulative effect of the test batteries is discussed and not the individual assessments, meaning it is hard to be certain what to attribute the predictive power to nor were the test batteries re-administered at later points to understand progression in different areas. To our knowledge, there have only been a few studies that have investigated the cognitive aptitude of SLI trainees throughout their studies (López Gómez et al., 2007; Macnamara and Conway, 2016; Stone, 2017). López Gómez et al. (2007) found that a nonsense-sign repetition test was a good predictor of successful Spanish Sign Language acquisition, whereas, for Stone’s cohort, the MLAT number-learning test was predictive of students’ BSL exam results. Both studies argued that these tasks directly or indirectly relate to how the phonological structure of signs is encoded. L2 sign language learners are known to struggle with phonological processing in the new visuospatial modality (e.g., Ortega and Morgan, 2015; Williams and Newman, 2016). This has also been shown in deaf signers who learn sign language as an L2 or late L1 and experience a ‘processing bottleneck’ at the phonological level (Mayberry and Fischer, 1989). Another study that has taken a re-test approach to cognition in SLI trainees is Macnamara and Conway (2016), who administered a battery of cognitive tests targeting WM capacity and SLI performance at four points throughout an ASL-English SLI training program. Their main findings were that WM capacity predicted initial SLI performance and that it was an even stronger predictor of final SLI performance. Additionally, students who performed well initially maintained a high level of performance, whereas those who performed poorly initially benefited more from the SLI training, but not enough to catch up to the higher level. Despite these initial longitudinal investigations into student SLI cognitive aptitude, none of these studies assessed students’ baseline skills before the start of their program, meaning that performance could have been already changed by sign language teaching or other factors.

### Cognitive adaptations from L2 sign learning

Research has shown that fluent signers outperform non-signers on several measures of visuospatial ability like mental rotation (MR) and image generation (for review, see Emmorey, 1998, 2002), suggesting skills-based enhancements from exposure to language in the visuospatial modality. Particularly, MR has been shown numerous times to be improved because of sign language experience (e.g., McKee, 1987; Talbot and Haude, 1993; Emmorey et al., 1998), indicating it is an important skill required for sign language use. As well as the need to mentally rotate to understand, e.g., topographical uses of signing space, Watkins et al. (2018) also suggest that MR skills are crucial to BSL comprehension when perceiving signs from the side, as opposed to a face-to-face orientation. Side-on comprehension is needed in many real-life situations, e.g., group conversations, or SLI scenarios, such as conferences, yet is often neglected in teaching materials and methods, where incidental side-on comprehension in class is relied upon, rather than being specifically instructed.

Some skill-based enhancements in visuospatial WM and MR extend into late L2 signers (e.g., Keehner and Gathercole, 2007; Kubicek and Quandt, 2021). However, like many interpreting aptitude studies, they lack baseline measures before sign learning or critical SLI instruction began. For example, Keehner and Gathercole found improved visuospatial WM in fluent late L2 signers working as BSL interpreters, but the authors acknowledge that their participants may simply have been spatially adept before learning to sign, which, in turn, may have facilitated successful L2 sign language acquisition. Thus, it is unclear whether such effects derive directly from signing experience, or whether those reaching fluency are predisposed to better cognitive abilities, such as MR or visuospatial WM. If pre-existing threshold visuospatial skills are found to be predictive of successful L2 sign language learning, these could then be targeted for specific training, either within a signing context or as a general cognitive skill, within SLI training programs. It has already been shown that deaf and hard of hearing children can improve their MR skills through targeted practice (Passig and Eden, 2001), which then feeds back into sign language fluency. An advantage of a longitudinal approach with a baseline measure at the start of the SLI program means we can detect both how skills progress across time, and how individual differences in baseline skills relate to this development.

### Present study and domains of investigation

Longitudinal studies are a good approach for investigating aptitude and related questions, as they allow the identification of developmental milestones and any individual differences in performance, as well as the time points at which learners begin to perform at the level of working interpreters.

One open question is the link between WM and modality in SLI (for further discussion, see also Wilson and Emmorey, 2003; Hall and Bavelier, 2011; Wang and Napier, 2013; Williams et al., 2015). Existing studies have not always distinguished between multimodal dual-attention WM tasks requiring both auditory and visuospatial attention, and unimodal WM tasks where only one modality must be attended to. Furthermore, most of the aforementioned research on SLI and WM only includes a single WM task in just one modality, and overall, very few studies have employed multimodal WM tasks. One exception is Bontempo and Napier (2009), who included a dual-task memory exercise (divided attention) in their pre-SLI-degree test battery, but they did not describe the results at a task level, only discussing the composite test battery. Here, we attempt to test three measures of WM: one auditory, one visuospatial, and one dual WM task with multimodal input to attend to (auditory and visuospatial) simultaneously (see Figure 1).

**FIGURE 1:** Example stills from the working memory tasks used in the study: **(A)** Dual *n*-back task (multimodal working memory, WM); **(B)** Corsi blocks task (visuospatial WM); **(C)** Digit span task (auditory WM).

To our knowledge, none of the existing studies on cognitive aptitude for SLI, whether based on students or working interpreters, have specifically looked at MR (despite being highlighted as a possible predictor by López Gómez et al. (2007), they did not include a rotation task in their test battery). Here we use two different tasks: one where 2D shapes simply need to be rotated in a circle (Figure 2A), and another that uses 3D-rendered blocks that must be rotated around the vertical axis only (Figure 2B). It is MR in this plane that should be the closest way the sign language input must be rotated while comprehended (Watkins et al., 2018).

**FIGURE 2:** Example stills from the two mental rotation (MR) tasks used in the study: **(A)** simple circular 2D shape rotation task showing an example “same” pair rotated 90°; **(B)** 3D-rendered block rotation task around vertical axis only, showing an example “mirror” pair rotated 150°.

We included two linguistic tasks that assess English skills. Initial English vocabulary knowledge was found to predict self-rated ASL proficiency after 1 semester of ASL instruction (Williams et al., 2017). English reading comprehension was also shown to improve during the SLI degree by Stone (2017), and we repeated the same measure here. Summarizing and paraphrasing are known to be an important skills in spoken language interpreting (e.g., Moser-Mercer, 1985; Russo and Pippa, 2004; Russo, 2014). Being able to comprehend and summarize complex spoken English before interpreting it into “chunks” of BSL is also required of SLI students and, thus, we created a task to assess this ability. We also include the MLAT Number Learning task used by Stone (2017) as a measure of phonological encoding, which was predictive of later BSL grades (see also Martinez and Singleton, 2019, who found sign learning and word learning to be highly correlated in hearing non-signers).

As Macnamara et al. (2011) pointed out, cognitive skills do not exist in a vacuum, and there has been a range of studies exploring SLI aptitude in terms of more social factors like disposition and personality (Stauffer and Shaw, 2006; Bontempo et al., 2014). Hence, we also include one personality measure of risk-taking that was predictive of continuation on the SLI degree in Stone (2017), the Barratt Impulsiveness Scale, version 11 (BIS-11; Patton et al., 1995). Specifically, Stone found that SLI students remaining in the degree program were significantly more impulsive, i.e., more likely to take risks than students who were rehoused in a Deaf Studies program (due to choice or poor BSL/interpreting exam performance). Macnamara et al. (2011) also found that a different measure of risk-taking (Behavioral Inhibition System; Carver and White, 1994) differentiated between highly skilled and less-skilled interpreters Lastly, we also used a non-verbal reasoning task as a control measure, which we do not predict will change over time, nor impact BSL or SLI performance.

This preliminary study asks three main research questions: (1) Do any of the cognitive and linguistic assessments predict being selected for, or continuing with, the SLI degree? (2) How do the cognitive and linguistic skills change throughout the SLI degree? (3) Are any of the cognitive or linguistic skills associated with BSL and SLI performance outcomes? In sum, we aim to see if we can replicate previous results in some domains by using identical or similar tasks as in previous longitudinal studies, as well as investigating some new areas (MR, and manipulating the modality of WM tasks). Taken together, these elements could help us get a step closer to understanding which cognitive and linguistic skills indicate the potential of an L2 sign language learner and a successful SLI student.

## Materials and methods

### Participants

Sign language interpreting students (*n* = 33) were recruited from two undergraduate degree programs: ‘MA (Hons) BSL (Interpreting, Translating and Applied Language Studies)’ at Heriot–Watt University (*n* = 23 total) or ‘BA (Hons) Interpreting (BSL/English)’ at the University of Wolverhampton (*n* = 10). Two consecutive year groups of Heriot-Watt students were tested (HW1: *n* = 11, HW2: *n* = 12; see Table 1). Across all cohorts, three participants were heritage signers of BSL and were, thus, excluded from later analyses. The remaining L2 participants mostly had only limited exposure to BSL before beginning their interpreting program (e.g., introductory courses). A further group of prospective candidates for the first HW cohort (HW0: *n* = 19) were tested at interview but were not selected for entry into the degree program. Therefore, data only exists for this group from session 1.

**TABLE 1:** Demographics of the cohorts of sign language interpreting (SLI) students who took part in the longitudinal study.

Institution	Heriot-Watt University			University of Wolverhampton
Cohort	Rejected	1st Cohort	2nd Cohort	Single cohort
Cohort code	HW0	HW1	HW2	WV
*N*	19	11	12	10
Mean age at session 1 (years; months)	24;2	22;8	27;1	26;3
Mean prior BSL exposure (years; months)	3;1	1;8	1;4	4;10
Session 1 (pre-course)	In-person	In-person	In-person	In-person
Session 2 (end of year 1)	NA	In-person	Online	Online
Session 3 (end of year 2)	NA	Online	Online	Online
Session 4 (midway year 3)	NA	NA	Online	Online

### Longitudinal study design

Participants were tested on a battery of cognitive and linguistic assessments at four sessions, approximately 1 year apart. Session one was before beginning the program and, thus, for most participants, before critical exposure to BSL had begun. Session two was at the end of the first year of the course, and the third session was at the end of the second year before students began their placement/internship years. The fourth and final session was halfway through this placement year. Due to disruption related to the COVID-19 pandemic (e.g., lack of equipment or suitable space for remote participation at home), as well as students dropping out of their courses or not being interested in further participation at later test sessions, it was not possible to re-test all participants at test sessions two to four. Furthermore, the online testing at later sessions was spread out more than planned compared to pre-pandemic testing, which was carried out in-person on specific dates at the Heriot-Watt and Wolverhampton University campuses.

### Description of test battery

First, the cognitive and linguistic aptitude assessments comprising the predictor variables are described, followed by the BSL and SLI assessments, which make up the outcome variables (see Table 2).

**TABLE 2:** All skills assessed in the longitudinal study and the test/re-test procedure by cohort.

Skill (assessment)	Session			
	Pre-degree	1st Year	2nd Year	3rd Year
	*n* = 33	*n* = 13	*n* = 11	*n* = 9
Multimodal WM (working memory; Dual *N*-Back)	All	All	All	HW2, WV
Visuospatial WM (Corsi Blocks)	All	All	All	HW2, WV
Auditory WM (Digit Span)	HW2, WV	–	HW2, WV	HW2, WV
2D MR (mental rotation; shape rotation)	HW1	HW1	All	HW2, WV
3D MR (block rotation)	HW2, WV	HW2, WV	All	HW2, WV
Phonological encoding (MLAT number learning)	HW2, WV	–	–	–
English comprehension (Kirklees reading)	All	All	All	–
Non-verbal reasoning (KBIT-2 matrices)	All	All	All	–
Summarizing (TED talk task)	HW2, WV	–	–	–
Impulsivity (Barratt Impulsiveness Scale)	–	–	All	HW2, WV
BSL sign repetition (copy-sign)	All	–	–	–
BSL sentence repetition (BSL-SRT)	NA	–	All	HW2, WV
BSL (BSL module grades)	NA	All	All	Placement
SLI (BSL to English task)	NA	NA	–	HW2, WV
SLI (English to BSL task)	NA	NA	–	HW2, WV
SLI (SLI module grades)	NA	NA	HW2, WV	Placement

#### Predictor variables

##### Working memory tasks

As a measure of multimodal WM, participants completed the Psychology Experiment Building Language (PEBL; Mueller, 2014; Mueller and Piper, 2014) test battery version of the dual *n*-back task (Jaeggi et al., 2008). In the task, participants must simultaneously recall a sequence of letters presented auditorily, as well as the spatial location of a sequence of squares, presented visually on a grid. Participants press a button when the letter or square location matches the letter or square location presented *n* trials ago. The task has one block each of 1-back, 2-back, and 3-back trials. The dependent measure was combined accuracy (average accuracy across both letter-matching and spatial matching).

For visuospatial WM, participants completed the PEBL version of the Corsi block-tapping task (Corsi, 1972; Kessels et al., 2000). In the task, participants must memorize the order, in which a sequence of blocks changes color and then click the blocks in the same order. The sequence gets progressively longer as the task goes on. The dependent measure was the number of correct responses.

As a measure of auditory WM, participants completed the PEBL test battery version of the Digit Span task (Croschere et al., 2012). In this task, participants must remember a sequence of numbers presented auditorily number-by-number, and then type in the sequence of numbers as it was heard. The sequence of numbers gets progressively longer as the task goes on. The dependent measure was the accuracy of responses.

##### Mental rotation tasks

At sessions one and two, HW1 participants completed the simple 2D PEBL MR task (Shepard and Metzler, 1988; Berteau-Pavy et al., 2011). The HW2 and WV groups also completed this task at sessions three and four. In this task, participants must decide if two shapes presented side-by-side on the screen are the same or different by mentally rotating them. The dependent measure was a speed-accuracy trade-off score that combines RT and accuracy measures, calculated using the Balanced Integration Score (Liesefeld et al., 2015; Liesefeld and Janczyk, 2019).

For 3D-MR, participants completed a 3D block rotation task comprising 96 three-dimensional stimuli validated by Ganis and Kievit (2015). The task was created using PsychoPy/Pavlovia (Peirce et al., 2022) and is freely available at https://pavlovia.org/freyawatkins/block_rotation. The task is a measure of MR around the vertical axis, where participants must decide whether two shapes presented side-by-side on the screen are identical or mirror images by mentally rotating them as quickly and accurately as possible. The dependent measure was again a speed-accuracy trade-off score, combining RT and accuracy into a single measure.

##### Phonological encoding

At session one, the HW2 and WV groups completed the Number Learning subtest of the MLAT (Carroll and Sapon, 1959; Carroll et al., 2010), which is a measure of “auditory alertness” and phonological encoding. Participants are taught a number system in a made-up language through auditory input and tested by being asked to translate new combinations of numbers from the made-up language back into English numerals. The test features 43 items. The dependent measure was response accuracy.

##### Linguistic tasks

As a measure of English reading comprehension, participants completed the revised Kirklees version of the Vernon Warden Reading Test (Warden, 1956; Hedderly, 1996). In the task, participants must complete 42 sentences by selecting the most appropriate word to fill a gap from the five options provided. Participants were given 10 min to complete the task, which was completed using pen and paper at face-to-face testing sessions and using a digitized version at online testing sessions. The dependent measure was test accuracy.

As a measure of summarizing ability, students had to listen to a short presentation (a TED talk on climate change and food, Ebi, 2019) and afterward suggest a title for the presentation and summarize the presentation in five key bullet points. The dependent measure was the accuracy of the summary.

##### Non-verbal reasoning

Participants completed the Matrices subtest from the Kaufman Brief Intelligence Test-2 (KBIT-2; Kaufman and Kaufman, 2004). In this task, participants are presented with visual stimuli with a specific rule or relationship, which participants must understand and then select the picture or pattern from the options provided that best fits that relationship or rule. Participants were given 10 min to complete the task, which was completed using pen and paper at face-to-face testing sessions and using a digitized version plus spreadsheet answer key at online testing sessions. The dependent measure was test accuracy.

##### Impulsivity

Participants completed the BIS-11 (Patton et al., 1995), a 30-item questionnaire, where they self-rate the frequency of their behavior and preferences regarding impulsivity. The dependent measure was the total score.

#### Outcome variables

##### British Sign Language performance

All students at session one completed a copy-sign task, which was a measure of BSL reception and production. The task consists of 10 BSL signs and three short BSL sentences, which were presented twice by a Deaf L1 signer and had to be reproduced by the students as accurately as possible. The accuracy of BSL production was coded by a sign language interpreter, with marks for phonological parameters (handshape, movement, location, orientation, and non-manual features) articulated correctly for individual signs, as well as phrasing and prosody for sentences.

At sessions three and four, students were tested on the BSL Sentence Reproduction Test (BSL-SRT; Cormier et al., 2012). The test involves viewing BSL sentences of increasing complexity and reproducing them as accurately as possible. The test is, therefore, an assessment of both BSL comprehension and production. Videos of BSL production were coded for accuracy by an SLI instructor, with one mark for each sentence reproduced correctly.

Module grades from BSL modules were collected from both semesters for the first 2 years of the course. For HW1 and HW2 students, grades included two first-year intensive practical modules in BSL and two second-year modules in Advanced BSL. For WV students, grades were made up of the first-year modules “Intermediate BSL Enhancement for Interpreters A, B, and C” and the second-year modules “Advanced BSL Enhancement for Interpreters A, B, and C”^1^. Third-year grades mostly relate to student placements and are not included in analyses. Grades follow the standard UK university grading system (0–100; whereby most marks fall between the range 40–80, see, e.g., Yorke et al., 2000).

##### Sign language interpreting performance

At session four, HW2 and WV participants completed two consecutive interpreting tasks hosted on GoReact (GoReact, 2022). In the first, they had to sequentially (not simultaneously) interpret a four-minute story from BSL into English. The story, signed by an L1 Deaf signer in an informal register, was about a COVID-19 vaccination appointment. In the second task, students interpreted a three-and-a-half-minute instructional video from English into BSL. In the video, a nurse with L1 English explains the procedure for visiting a COVID-19 ward in a hospital, using a more formal register. Students were allowed to pause the video to ‘chunk’ their interpretation as they saw fit: this ‘chunking’ skill was also part of the assessment of the interpretation. These tasks were assessed by an SLI educator and graded like university assignments (0–100). The total score for each consecutive interpreting task was calculated based on poise, style, consecutive management, comprehension, conceptual rendition, vocabulary, accuracy, repairs, and an overall mark.

Module grades from second-year interpreting modules were also collected. For HW1 and HW2 students, these comprised the ‘Introduction to Translation and Interpreting skills’ module, while for WV students, the modules ‘Consecutive Interpreting 1 and 2’. Third-year grades mostly relate to student placements and are not included in analyses.

### Ethics approval statement

For the initial cohort (HW0 and HW1), ethical approval was gained from Heriot-Watt University. For the HW2 and WV cohorts, approval was gained from the University of Birmingham Science, Technology, Engineering, and Mathematics Ethical Review Committee (ERN_18-1170). Updated ethical approval was gained for later testing sessions, which took place online due to the COVID-19 pandemic. All subjects gave written informed consent in accordance with the Declaration of Helsinki, as well as video consent for tasks where participants were filmed while signing.

### Test procedure

Within each testing session, the order of assessments was randomized. This was dependent in part on the availability of researchers to run an assessment at any given time and on computer availability for online testing.

### Statistical analysis

#### Analysis plan

Our exploratory analyses are divided into three sections. First, we use stepwise backward logistic regression to determine whether any assessments were predictive of (1) being selected for, and (2) continuing with the SLI degree. The second analysis examines changes in the linguistic and cognitive assessments over time, looking at each predictor in turn. Here we use linear mixed models with random effects structure for participants per task, with initial BSL proficiency as a covariate. Finally, the third analysis looks at correlations between the linguistic/cognitive assessments and (1) BSL performance and (2) SLI performance (grades and BSL/SLI tasks). Here, we begin by examining whether there are any relationships between the predictors at the pre-degree initial testing session and later outcome variables, and then looking at any relationships when assessments are repeated at later testing points. We calculate *r*^2^ values and also fit linear mixed models with initial BSL proficiency as a covariate.

#### Data availability and reproducibility

We report all data exclusions (if any), all manipulations, and all measures in the study, and we attempt to follow JARS (Kazak, 2018). This study’s design and its analyses were not pre-registered. In line with standards of reproducible research, the scripts, and data (excluding video data and possibly identifying variables, such as age) are made available with this publication and can be retrieved on the following publicly accessible repository: https://osf.io/kjctg. We used R version 4.0.5 (R Core Team, 2021) plus the packages {lme4} v1.1.27.1 (Bates et al., 2015), {sjPlot} v2.8.10 (Lüdecke, 2021) and {blorr} v0.3.0 (Hebbali, 2020) for the regression/mixed-effects model analyses and output reported below, plus {effsize} v0.8.1 (Torchiano, 2020) to calculate effect sizes. For data processing and visualization, we used the package {tidyverse} v1.3.1 (Wickham et al., 2019), for file organization {here} v1.01 (Müller, 2020), and for plotting details we used {scales} v1.1.1 (Wickham and Seidel, 2020), {PupillometryR} v0.0.3 (Forbes, 2020), {sdamr} v0.1.0 (Speekenbrink, 2021), {plotrix} v3.8.1 (Lemon, 2006), and {patchwork} v1.1.1 (Pedersen, 2020).

#### Attrition and missing data

Our longitudinal study was subject to high levels of attrition over time, for a combination of known and unforeseen reasons. The aforementioned high drop-out rate from SLI degree programs was a known factor that we expected would greatly reduce participation at later sessions. Missing data from these participants could be considered ‘missing-at-random’, where degree program drop-out relates to poor grades or difficulty with the content of the program. However, the outbreak of the COVID-19 pandemic introduced a large number of reasons for data to be ‘missing-not-at-random’, which we could not account for with auxiliary variables (e.g., socioeconomic background, income-to-needs ratio, participant disability, parental education). For example, the pandemic necessitated online testing at sessions 2, 3, and 4. This was not equally accessible to all participants, due to differences in access to equipment, technological knowledge, time, space to participate remotely, etc. Furthermore, pandemic-related illness also prevented some participants from repeating tasks at specific time points. While multiple imputation of missing data is possible, even when data are missing-not-at-random for reasons like these (see, e.g., Madley-Dowd et al., 2019), this approach is only considered appropriate when auxiliary variables that may have correlated with missingness are also present in the dataset. Since we did not collect initial data on these factors, imputing missing data would not have produced less biased estimates.

## Results

### Predictors of selection and remaining in sign language interpreting degree program

#### Predictors of selection

The first sub-analysis examines whether any of the cognitive and linguistic assessments at session one (pre-degree) were predictive of being selected for the degree program, using data from the HW1 cohort, plus the candidates who were assessed at the interview but not selected (HW0). We fit a backward stepwise logistic regression model to identify possible predictors of the binary outcome variable “selected” (0, 1) out of the following predictor variables: multimodal WM, visuospatial WM, non-verbal reasoning, English vocabulary, 2D-MR, and initial BSL self-rating. At each step, variables were chosen based on *p*-values, and a default *p*-value threshold for backward stepwise regression of 0.1 was used to set a limit on the total number of variables included in the final model. The stepwise regression reduced the predictors to just the 2D-MR score (*z* = 1.78, *p* = 0.075) and BSL self-rating (*z* = 1.91, *p* = 0.056), whereby higher 2D-MR scores and higher BSL self-ratings, respectively, were both significant predictors of being selected for the degree. While we did not have enough data from the copy-sign task coded to include in the model, self-rated BSL proficiency and copy-sign task scores were significantly positively correlated (*r*^2^ = 0.42, *t* = 3.16, *p* = 0.007).

#### Predictors of continuation

Our second sub-analysis looks at students across the three cohorts who were selected for the degree program, i.e., excluding those who were not successful in gaining a place at the interview. Here, we ask whether any of the initial assessments carried out pre-degree predicted whether students were continuing with the degree program at the time of writing (in their final or penultimate year). Again, we fit a backward stepwise logistic regression model to identify possible predictors of the binary outcome variable “continuing” (0, 1) out of the following predictor variables: multimodal WM, visuospatial WM, non-verbal reasoning, English vocabulary, and initial BSL self-rating. At each step, variables were chosen based on *p*-values, and a default *p*-value threshold for backward stepwise regression of 0.1 was used to set a limit on the total number of variables included in the final model. The stepwise regression reduced the predictors of continuing with the SLI degree to just visuospatial WM (*z* = –1.77, *p* = 0.078), whereby a higher visuospatial WM score significantly predicted continuing on the degree. As an additional analysis, we also modeled impulsivity at the end of the second year, but this did not predict continuation in the degree.

### Changes in cognitive and linguistic skills during sign language interpreting program

In our second set of analyses, we look at all the cognitive and linguistic assessments in turn and examine their change over time, as students progress through the SLI program. All linear models have initial BSL skill as a covariate and random effects for participants, and use a standard *p*-value threshold for linear models of 0.05. Models of English comprehension also included age at the initial testing session as a covariate.

#### Working memory tasks over time

Multimodal WM (Dual N-Back) was significantly improved after 2 years of study compared to pre-degree (*t* = 2.32, *p* = 0.02, *d* = 0.56; Figure 3A). However, this improvement did not hold in the final session (*t* = 0.12, *p* = 0.91) compared to pre-degree.

**FIGURE 3:** Changes in sign language interpreting student performance on four cognitive assessments over time: **(A)** multimodal working memory (WM) was significantly improved after 2 years of study compared to pre-degree (*t* = 2.32, *p* = 0.02, *d* = 0.56); **(B)** visuospatial WM was significantly improved after 1 year of study compared to pre-degree (*t* = 2.01; *p* = 0.044, *d* = 0.29); **(C)** auditory WM was significantly improved after 3 years of study compared to pre-degree (*t* = 2.72, *p* = 0.007, *d* = 1.57); **(D)** 3D mental rotation (MR) was significantly improved compared to pre-degree at all subsequent sessions (vs. first year: *t* = 2.51, *p* = 0.012, *d* = 1.32; vs. second-year: *t* = 4.6, *p* < 0.001, *d* = 0.91; vs. third-year: *t* = 5.31, *p* < 0.001, *d* = 1.68).

Performance on the visuospatial WM task (Corsi Blocks) was significantly improved after 1 year of study compared to pre-degree (*t* = 2.01; *p* = 0.044, *d* = 0.29; Figure 3B). However, this improvement did not hold for the latter two sessions (second year: *t* = –0.06, *p* = 0.95; third year: *t* = 1.52, *p* = 0.13).

Auditory WM performance (Digit Span) was not significantly improved by the second year compared to pre-degree (*t* = 0.53, *p* = 0.59), but third year accuracy was significantly higher than pre-degree (*t* = 2.72, *p* = 0.007, *d* = 1.57; Figure 3C).

#### Mental rotation tasks over time

Performance on the 2D shape rotation task was significantly improved after 1 year of study compared to pre-degree (*t* = 2.71, *p* = 0.007)^2^. Interestingly, the covariate initial BSL skill played a negative role in predicting 2D-MR performance overall (*t* = –2.21, *p* = 0.028). Reaction times were significantly faster than pre-degree at all subsequent sessions (first year: *t* = –3.9, *p* < 0.001, *d* = 1.07; second year: *t* = –2.88, *p* = 0.004; third-year: *t* = –3.32, *p* = 0.001). On the 3D block rotation task, speed-accuracy trade-off scores were significantly higher than pre-degree at all subsequent sessions (first year: *t* = 2.52, *p* = 0.012, *d* = 1.32; second year: *t* = 4.6, *p* < 0.001, *d* = 0.91; third year: *t* = 5.31, *p* < 0.001, *d* = 1.68; Figure 3D). Likewise, reaction times on the 3D-MR task were significantly faster than pre-degree at all subsequent sessions (first year: *t* = –2.2, *p* = 0.028, *d* = 1.97; second-year: *t* = –5.3, *p* < 0.001, *d* = 1.33; third year: *t* = –5.69, *p* < 0.001, *d* = 2.53), although accuracy alone was only significantly improved at the final session (*t* = –2.16, *p* = 0.031, *d* = 0.57).

#### Linguistic and other assessments over time

English reading comprehension (Kirklees) showed no effect of testing session when comparing pre-degree accuracy to first-year performance (*t* = –1.19, *p* = 0.24) or second-year performance (*t* = 1.38, *p* = 0.17). Our control measure, non-verbal reasoning (KBIT-2 Matrices), also showed no effect of session when comparing pre-degree accuracy with first-year performance (*t* = –1.28, *p* = 0.20) or second-year performance (*t* = 0.5, *p* = 0.62). Impulsiveness (BIS) was only tested during the second and third years but was significantly reduced at the final testing session compared to the penultimate session (*t* = –2.39, *p* = 0.017, *d* = 0.28), though the effect size was small. Due to time constraints on in-person testing and limited data from online testing sessions, the tasks assessing phonological encoding and summarizing were only conducted at one session each, and, therefore, no change-over-time analyses were conducted.

### Predictors of British Sign Language and sign language interpreting performance

Our final set of analyses examines whether any of the cognitive and linguistic assessments were associated with (1) BSL and (2) SLI performance. Firstly, we look at whether any assessments were related to BSL measures, such as grades in BSL modules and BSL Sentence Reproduction Test scores. Due to the high level of attrition across the longitudinal study, we do not attempt to fit a large mixed model with all predictors for outcome variables at the final session. Instead, we report correlations and individual regression analyses, modeling BSL and SLI measures as a function of predictor assessments, with initial BSL proficiency as a covariate. Models of English comprehension also include age at the initial testing session as a covariate.

#### Working memory tasks and British Sign Language performance

As a reminder of our hypotheses: we did not predict that the WM assessments would have an impact on any BSL outcomes, other than visuospatial WM. There was no relationship between initial multimodal WM (Dual N-Back) and second year BSL grades (*r*^2^ = 0.006), nor did multimodal WM relate to third-year BSL-SRT scores (*r*^2^ = 0.002). The relationship between third-year multimodal WM skill and SRT scores was not significant (*r*^2^ = 0.12, *t* = 0.83, *p* = 0.44). We found no relationship between initial visuospatial WM (Corsi Blocks) and second-year BSL grades (*r*^2^< 0.001), nor with third-year BSL-SRT scores (*r*^2^ = 0.10). However, third-year SRT scores were significantly positively associated with visuospatial WM skill in second-year (*r*^2^ = 0.609, *t* = 2.73, *p* = 0.041; Figure 4A), but the positive correlation with third-year WM was not significant (*r*^2^ = 0.301, *t* = 1.55, *p* = 0.17; Figure 4B). In terms of auditory WM, initial digit span scores were not associated with first (*r*^2^ = 0.12) or second-year BSL grades (*r*^2^ = 0.14), nor with third-year BSL-SRT scores (*r*^2^ = 0.001).

**FIGURE 4:** Correlations between sign language interpreting (SLI) student performance on working memory tasks and British Sign Language (BSL) measures: **(A)** second-year visuospatial working memory (WM) was a significant predictor of third-year BSL-SRT scores (*n* = 7; *r*^2^ = 0.609, *t* = 2.73, *p* = 0.041); **(B)** third-year visuospatial WM was positively correlated with third-year BSL-SRT scores, but this relationship was insignificant (*n* = 9; *r*^2^ = 0.301, *t* = 1.55, *p* = 0.17).

#### Mental rotation tasks and British Sign Language performance

There was no relationship between performance on the initial 2D rotation task and second-year BSL grades (*r*^2^ = 0.001). The relationships between second-year 2D-MR scores and second-year BSL grades (*r*^2^ = 0.27, *t* = 1.64, *p* = 0.14), as well as between third-year rotation scores and third-year BSL-SRT scores (*r*^2^ = 0.19, *t* = 1.5, *p* = 0.18), showed moderate positive correlations, but these were also not significant.

Likewise, for 3D-MR, there was no relationship between initial 3D rotation skill and second-year BSL grades (*r*^2^< 0.001). Initial 3D-MR scores were positively correlated with third-year BSL-SRT scores, but this correlation was not significantly different from zero (*r*^2^ = 0.37; *t* = 1.81, *p* = 0.12; Figure 5A). Second-year 3D-MR and second-year BSL grades were also strongly correlated, but the effect was marginally insignificant (*r*^2^ = 0.39, *t* = 2.21, *p* = 0.054; Figure 5B). Third-year 3D rotation scores were unrelated to third-year BSL-SRT scores (*r*^2^ = 0.12).

**FIGURE 5:** Correlations between sign language interpreting (SLI) student performance on mental rotation (MR) tasks and British Sign Language (BSL) measures: **(A)** pre-degree 3D-MR skill was positively correlated with third-year BSL-SRT scores, but this relationship was not significant (*n* = 9; *r*^2^ = 0.37; *t* = 1.81, *p* = 0.12); **(B)** second-year 3D-MR was positively correlated with second-year BSL grades, but this relationship was marginally insignificant (*n* = 12; *r*^2^ = 0.39, *t* = 2.21, *p* = 0.054).

#### Linguistic and other assessments and British Sign Language performance

There was a significant positive relationship between initial English reading comprehension (Kirklees) and first-year BSL grades (*r*^2^ = 0.19, *t* = 2.90, *p* = 0.008; Figure 6A), but not with subsequent BSL grades (*r*^2^ = 0.02). The relationship between initial reading comprehension and third-year BSL-SRT score showed a moderate positive correlation, but this was not significant (*r*^2^ = 0.237, *t* = 1.56, *p* = 0.17; Figure 6B). In terms of the summarizing task, as predicted, there was no impact on first- (*r*^2^ = 0.002) or second-year BSL grades (*r*^2^ = –0.06), nor was there a relationship with third-year BSL-SRT score (*r*^2^ = 0.01).

**FIGURE 6:** Correlations between initial sign language interpreting (SLI) student performance on English reading comprehension and later British Sign Language (BSL) measures: **(A)** pre-degree English comprehension was a significant predictor of first-year BSL grades (*n* = 29; *r*^2^ = 0.19, *t* = 2.90, *p* = 0.008); **(B)** pre-degree English comprehension was moderately positively correlated with third-year BSL-SRT scores, but this relationship was not significant (*n* = 9; *r*^2^ = 0.237, *t* = 1.56, *p* = 0.17).

We found no relationship between initial phonological encoding ability (MLAT Number Learning) and second-year BSL grades (*r*^2^ = 0.033), nor was there a relationship with third-year BSL-SRT score (*r*^2^< 0.001). There was no association between impulsivity (BIS) and second-year BSL grades (*r*^2^ = 0.009). Impulsivity had a slight negative correlation with third-year BSL-SRT scores, but this relationship was not significant (*r*^2^ = –0.27, *t* = –1.45, *p* = 0.19). There was no relationship between our control measure (non-verbal reasoning; KBIT-2 Matrices) and second-year BSL grades (*r*^2^ = 0.001). Non-verbal reasoning also did not correlate with third-year BSL-SRT scores (*r*^2^ = 0.004).

Now we turn to look at the relationships between cognitive and linguistic assessments and measures of SLI performance, such as SLI module grades and the two final consecutive SLI tasks.

#### Working memory tasks and sign language interpreting performance

There was no significant relationship between initial multimodal WM scores and second-year interpreting grades (*r*^2^ = 0.11), nor with performance on the third-year English-to-BSL consecutive interpreting task (*r*^2^ = 0.12). This correlation was slightly stronger for third-year multimodal WM scores, but, again, not significantly so (*r*^2^ = 0.16, *t* = 0.7, *p* = 0.51). Initial multimodal WM did not affect scores on the consecutive interpreting task from BSL to English (*r*^2^ = 0.06).

In terms of visuospatial WM, there was no link between initial performance on the Corsi Blocks task and second-year interpreting grades (*r*^2^ = 0.008), nor did a relationship emerge with visuospatial WM at later testing sessions. There was a stronger yet insignificant correlation between initial visuospatial WM and scores on the third-year English-to-BSL consecutive interpreting task (*r*^2^ = 0.29, *t* = 1.27, *p* = 0.25), and for second-year visuospatial WM, this relationship was only marginally insignificant (*r*^2^ = 0.57, *t* = 2.48, *p* = 0.056; Figure 7A). Second-year visuospatial WM was also positively correlated with performance in the third-year consecutive interpreting task from BSL to English, but, again, the correlation was insignificant (*r*^2^ = 0.46, *t* = 1.82, *p* = 0.14).

**FIGURE 7:** Correlations between sign language interpreting (SLI) student performance on working memory (WM) tasks and SLI measures: **(A)** Second-year visuospatial WM skill was positively correlated with performance on the third-year English-to- British Sign Language (BSL) interpreting task, however, this relationship was marginally insignificant (n = 8; *r*^2^ = 0.57, *t* = 2.48, *p* = 0.056); **(B)** pre-degree auditory WM was correlated with 2nd-year SLI grades but this relationship was marginally insignificant (*n* = 13; *r*^2^ = 0.24; *t* = 1.96, *p* = 0.076).

There was a promising positive correlation between initial auditory WM (Digit Span) scores and SLI grades in the second year, which was marginally insignificant (*r*^2^ = 0.24 *t* = 1.96, *p* = 0.076; Figure 7B). Auditory WM at the final testing session was not related to the final English-to-BSL consecutive interpreting task (*r*^2^ = 0.12), nor the BSL-to-English task (*r*^2^ = 0.03).

#### Mental rotation tasks and sign language interpreting performance

There was no relationship between initial 2D-MR skill and second-year SLI grades (*r*^2^ = 0.038). We found stronger correlations between second-year SLI grades and 2D-MR skills in both second year (*r*^2^ = 0.24, *t* = 1.64, *p* = 0.14) and third-year (*r*^2^ = 0.39, *t* = 2.91, *p* = 0.027), the latter was statistically significant. For the English-to-BSL consecutive interpreting task, there were small positive correlations with second-year (*r*^2^ = 0.2) and third-year 2D-MR (*r*^2^ = 0.18), but these were not significant. However, for the third-year BSL-to-English interpreting task, the relationship with 2D-MR was stronger: second-year 2D-MR skill was a significant predictor (*r*^2^ = 0.6, *t* = 2.95, *p* = 0.042; Figure 8A) while third-year 2D-MR skill was a marginally insignificant predictor (*r*^2^ = 0.31, *t* = 2.11, *p* = 0.088; Figure 8B).

**FIGURE 8:** Correlations between sign language interpreting (SLI) student performance on mental rotation (MR) tasks and SLI measures: **(A)** second-year 2D-MR was a significant predictor of scores on the third-year British Sign Language (BSL)-to-English interpreting task (*n* = 7, *r*^2^ = 0.6, *t* = 2.95, *p* = 0.042); **(B)** third-year 2D-MR was correlated with scores on the third-year BSL-to-English interpreting task, but this relationship was marginally insignificant (*n* = 8, *r*^2^ = 0.31, *t* = 2.11, *p* = 0.088); **(C)** pre-degree 3D-MR was positively correlated with scores on the third-year English-to-BSL interpreting task, but this relationship was not significant (*n* = 9, *r*^2^ = 0.27, *t* = 1.32, *p* = 0.24); **(D)** pre-degree 3D-MR was correlated with scores on the third-year BSL-to-English interpreting task, but this relationship was marginally insignificant (*n* = 8, *r*^2^ = 0.48, *t* = 2.004, *p* = 0.101).

For 3D-MR, there was a moderate yet insignificant positive correlation between initial rotation skill and second-year interpreting grades (*r*^2^ = 0.24). This correlation became stronger over time (vs. second-year 3D rotation: *r*^2^ = 0.31; vs. third-year 3D rotation: *r*^2^ = 0.54, *t* = 2.85, *p* = 0.029), the latter relationship being significant. Initial 3D-MR also had a moderate but insignificant positive correlation with third-year English-to-BSL consecutive interpreting performance (*r*^2^ = 0.27, *t* = 1.32, *p* = 0.24; Figure 8C), although there was no correlation with later 3D-MR scores. Initial 3D-MR skill was also positively correlated with third-year consecutive interpreting from BSL to English, and this relationship was marginally insignificant (*r*^2^ = 0.48, *t* = 2.004, *p* = 0.101; Figure 8D). However, this correlation got weaker over time (vs. second-year 3D rotation: *r*^2^ = 0.29; vs. third-year 3D rotation: *r*^2^ = 0.16).

#### Linguistic and other assessments and sign language interpreting performance

There was no relationship between English sentence reading (Kirklees) at any time point and SLI grades, or with either of the consecutive SLI tasks. There was also no link between the pre-degree summarizing task and second-year SLI grades (*r*^2^ = 0.002), nor with either interpreting task.

We also found no significant relationship between non-verbal reasoning (KBIT-2 Matrices) and any SLI measures. There was no relationship between impulsivity (BIS) and SLI grades. There was a slight negative correlation between impulsivity and English-to-BSL consecutive interpreting, as well as between impulsivity and the consecutive interpreting task from BSL to English (*r*^2^ = –0.27), however, these were not significant.

#### Correlations among measures of British Sign Language and sign language interpreting performance

Second-year SLI grades were significantly correlated with both first-year BSL grades (*r*^2^ = 0.68, *t* = 7.21, *p* < 0.001) and second-year BSL grades (*r*^2^ = 0.69, *t* = 6.79, *p* < 0.001). The initial copy-sign task was a marginally insignificant predictor of first-year BSL grades (*r*^2^ = .46, *t* = 2.25, *p* = 0.054), but not second-year BSL grades (*r*^2^ = 0.21, *t* = 0.84, *p* = 0.43). Interestingly, the initial copy-sign task had a stronger correlation with SLI grades in the second year (*r*^2^ = 0.36, *t* = 2.08, *p* = 0.076) than with second-year BSL grades, but again this was marginally insignificant. Performance on the third-year BSL-SRT task was significantly correlated with first-year BSL grades (*r*^2^ = 0.66, *t* = 3.37, *p* = 0.015) and strongly correlated with second-year BSL grades (*r*^2^ = 0.53, *t* = 2.25, *p* = 0.074), which was a marginally insignificant predictor. The two consecutive SLI tasks (BSL-to-English and English-to-BSL) were also significantly correlated with each other (*r*^2^ = 0.79, *t* = 4.14, *p* = 0.009).

## Discussion

### Summary of key findings

In this exploratory study, we saw several significant relationships between cognitive and linguistic skills and SLI degree program outcomes. Firstly, we found that 2D-MR skill and initial self-rated BSL proficiency were significant predictors of selection for the SLI degree, whereas visuospatial WM predicted the continuation of the course. Next, we examined the impact of the SLI degree program on cognitive and linguistic skills over time, by first collecting baseline measures of these skills and repeating testing at three further sessions. We found improvements in multimodal WM by the end of the second year of the degree, in visuospatial WM by the end of the first year, and in auditory WM by the final testing session in the third year. While multimodal and visuospatial WM did not remain at these improved levels at subsequent sessions, both 2D- and 3D-MR skills were improved by the first year of the degree and consistently remained at these higher levels throughout our longitudinal study. In terms of cognitive and linguistic predictors of later BSL and SLI task performance, there were several significant and marginally insignificant results of note, despite our small sample size. First-year BSL grades were significantly predicted by pre-degree English comprehension; second-year BSL grades were strongly correlated with second-year 3D-MR (marginally insignificant), and third-year BSL-SRT scores were significantly predicted by second-year visuospatial WM. Second-year visuospatial WM was also strongly correlated with scores on the English-to-BSL interpreting task, and pre-degree auditory WM was strongly correlated with second-year SLI grades (both marginally insignificant). In terms of the third-year BSL-to-English interpreting task, 3D-MR was a significant or marginally insignificant predictor at three different testing sessions (pre-degree, second year, and third year). We now turn to consider some issues with data collection and attrition, and then move on to a detailed discussion of each of our three research questions and their related analyses in turn.

### Issues with data collection and attrition

The various effects of the COVID-19 pandemic had a considerable impact on our exploratory study, mostly in terms of student withdrawals from the degree program and the difficulties of re-testing students online at later sessions, making it more of a preliminary investigation. In particular, the earliest cohort (HW1), for whom the practical placement year fell during the first year of the pandemic, was affected heavily by withdrawals. Only a minority remained in the SLI degree program by the final year (just three of the original 12, i.e., 25%; one student joined the year group below). Some of those who withdrew continued on a BSL-only program, while others switched to unrelated degree courses or left university altogether. Anecdotal evidence from program instructors and students themselves suggests that the main reason for the high-withdrawal rate in this cohort was indeed the various impacts of the pandemic, which our statistical models had no way to account for without further demographic auxiliary variables. In particular, having to do interpreting placements remotely seemed to be isolating and discouraging for students, and not the immersive experience it might have been in-person. As a result, it is likely that capable and otherwise potentially successful students (particularly in this cohort) ended up withdrawing from their SLI program. However, it should be noted that most students in the other two cohorts remained in their programs. We believe our data still offer valuable insights about SLI aptitude given the range of assessments tested across multiple sessions, given the present lack of longitudinal work with baseline measures in the literature.

### Predictors of selection and remaining in sign language interpreting degree program

In our initial analyses, we saw some limited evidence of initial pre-degree assessments predicting whether students were either selected for or continued with, their SLI degree program. For the selection analysis, the best predictors were initial self-rated BSL proficiency and the 2D-MR task. Unsurprisingly, those students with some initial signing proficiency were more likely to be selected ahead of those with no knowledge of BSL and deaf culture. However, this could also be an indicator of confidence, and there may be an unconscious selection bias for students who appear more confident. This result also highlights that it is difficult to test SLI aptitude in university students from a complete baseline of no BSL exposure at all, since many are unlikely to commit to a degree without some prior signing experience. Furthermore, in recent years there have been greater opportunities to start learning BSL in secondary schools than has historically been the case. Although timing and funding constraints meant we were not able to code enough of the copy-sign data to include it as a predictor in the selection model, the data, available suggest that scores on the task correlated significantly with applicants’ BSL proficiency self-ratings. While our copy-sign task featured real BSL signs, many of our participants would not yet have been familiar with all the signs used. In this sense, it is similar to the nonsense sign repetition tasks used by López Gómez et al. (2007) and Stone (2017), which also involved phonological encoding and perceptuo-motor skills and were found to be good predictors of later success in their cohorts. The 2D-MR task was also a good predictor of selection, and this is an interesting result given other strong correlations between initial 3D-MR performance and later outcome measures. However, our selection analysis was conducted on just two cohorts (HW0 and HW1) and only five assessments, mostly due to time constraints at the interview stage (latter cohorts were tested during the first week of term, which meant we could test more assessments in a less stressful environment for participants). Future studies could aim to measure other skills at the initial interview stage, which could not be included here due to practical constraints. In particular, 3D-MR and auditory WM would be good candidates, since we found evidence that pre-degree performance in both of these domains in our other cohorts was strongly correlated with third-year SLI performance and SLI grades, respectively. This also suggests that an intervention study that targets improving these general cognitive skills before SLI specialization might be instructive. Lastly, it should be reiterated that SLI program instructors did not have access to the data from the initial assessment session when deciding whether to accept applicants to their degree programs.

In the continuation analysis, there was a significant relationship between pre-degree visuospatial WM and remaining on the SLI degree, whereby higher visuospatial WM scores were associated with continuation. One interpretation of this result is that the cognitive demands of signing and interpreting in the new visuospatial modality are possibly a factor that (consciously or unconsciously) makes students more likely to withdraw from the program (see, e.g., Grbić, 2009). Due to the high withdrawal rate in one specific cohort, it was not possible to include a MR task in the selection model since different cohorts did different rotation tasks in the first session. However, it would be interesting to see whether other cognitive tasks involving visuospatial cognition are also associated with program drop-out, such as the copy-sign task. In terms of impulsivity, we did not replicate the result seen by Stone (2017), whereby the BIS predicted continuation on the SLI degree vs. switching to a Deaf Studies course. Due to testing session time constraints, we only introduced the BIS from session 3 onward, where all testing was already online due to the pandemic, but ideally, we would have also taken a baseline measure of risk-taking. It is quite likely that our participants’ usual risk aversion strategies and levels of impulsiveness were inhibited or changed by the ongoing pandemic. The potential for impulsiveness to impact learning behaviors (e.g., having the confidence to attend deaf social events to practice BSL, etc.) was greatly restricted due to pandemic-related safety measures. In future larger studies that follow students through to graduation and beyond, it would be interesting to see whether specific cognitive and linguistic skills are associated with continuation or drop-out at particular points in time; for example, during placements, or once students start interpreting modules.

### Changes in cognitive and linguistic skills during sign language interpreting program

In terms of changes in cognitive and linguistic skills throughout the degree, there was evidence of improvement in several domains. All three WM tasks (multimodal, visuospatial, and auditory) showed some signs of improvement across testing sessions, although performance did not remain at this higher level. Visuospatial WM (Corsi Blocks) and multimodal WM (Dual N-Back) were improved by timepoints two and three, respectively, but these changes did not hold to the final session, nor was there any further improvement. These results are harder to interpret, but it could be that these regressions are related to reduced opportunities to practice BSL and SLI skills at certain points in the degree program. This is likely to have been the case at later sessions due to the effects of the COVID-19 pandemic. Alternatively, these regressions may be explained by the varying demands of the SLI degree program tapping into different aspects of WM more frequently at different time points during the course. Auditory WM (Digit Span) was only at a higher level at the final testing session, midway through the placement year, suggesting there may be potential for further improvement beyond our study yet within the SLI degree. Further testing through to degree completion could be instructive here, as most of our predictions regarding WM were related to SLI, and not BSL learning. In the first 2 years of the SLI program, the focus is mostly on acquiring BSL, where there is a greater emphasis on visuospatial skills, before beginning to interpret. Since the students do much more SLI in their placement year and final year, we would expect the greater potential for this to feedback into WM skills only toward the end of the degree, and beyond during professional practice.

As hypothesized, MR ability in SLI students improved over time, which fits with a wide body of literature on improved visuospatial cognition through sign language use (e.g., McKee, 1987; Talbot and Haude, 1993; Emmorey, 1998; Emmorey et al., 1998; Keehner and Gathercole, 2007; Kubicek and Quandt, 2021). In particular, the improvements on the 3D-MR task between the pre-degree and the final session had the strongest effect size across the entire longitudinal study. Results in the 2D-MR task were less clear-cut, with improved performance by the second session followed by a regression at later sessions in terms of speed-accuracy trade-off alone, but faster reaction times by both the second- and third-year sessions compared to the initial testing session. However, as suggested by Watkins et al. (2018), it is the rotation around the vertical axis, as assessed by the 3D block rotation task, which should most closely resemble the plane in which sign language input must be rotated during language processing. The 2D-MR task used here involved simple circular rotation, which does not map as clearly onto any visuospatial transformations during BSL use. In this sense, it is unsurprising that greater improvements over time were seen in the 3D-MR task and not the 2D-MR task, in tandem with L2 BSL learning during the degree program. The stronger improvement in the 3D-MR task involving rotation around the vertical axis, which is required during sign comprehension to understand someone signing from a different viewing angle; for example, provides some evidence that it is experienced with rotation in this plane through BSL practice, which is driving the improvement in 3D-MR, and not other types of rotation (e.g., signs that move from a palm-up to palm-down orientation). This also suggests that explicitly targeting improvement in comprehending sign language input from various angles would be beneficial.

For English reading comprehension, we did not see the same improvement over time as in Stone (2017), where Kirklees scores were significantly better by the end of the third year versus the start of the first year. Due to time constraints during testing, we could not repeat this task at our final third-year testing session. We assessed it for the final time at the end of the second year, which may be why we could not replicate this result. However, the Kirklees scores of our SLI students at the end of the second year were just below the level of Stone’s third-year students, who, in turn, scored significantly lower than the working BSL-English interpreters who were also tested. Given the lack of improvement in this preliminary study and the conclusion of Stone (2017), it may be that experience working as an interpreter improves English skills (perhaps due to exposure to a wider range of vocabulary during interpreting), above and beyond any improvement seen during a university degree program. Age is generally a reliable predictor of vocabulary size (e.g., Ben-David et al., 2015), with better vocabulary scores as age increases. While it was not a significant covariate in this study, our sample of university students unsurprisingly did not have an even spread of our ages (two-thirds of our participants were aged 23 or under when the course began).

### Predictors of British Sign Language and sign language interpreting performance

There were several strong correlations between the cognitive/linguistic skills assessed and measures of BSL and SLI performance, some of which were statistically significant.

Starting with BSL outcomes, first-year BSL grades were significantly predicted by English reading comprehension, a correlation that was particularly strong for those with lower English and lower BSL scores (Figure 3A). This suggests that weaker English skills at the start of an SLI program may initially be a hindrance to L2 language learning in a new modality. However, SLI students who perform poorly in English initially seem to catch up by later testing sessions, by which point English comprehension was no longer predictive of BSL performance, which might be a consequence of exposure to English use in a university setting. Second-year BSL grades were correlated positively with 3D-MR skills in the same year, which fits with studies showing that MR improves gradually in line with sign language learning and does not just improve once sign language fluency is reached (Kubicek and Quandt, 2021). Interestingly, however, there was also a promisingly strong correlation, albeit not significant, between initial 3D-MR and third-year BSL-SRT scores (Figure 5A). This suggests that at least some of the success in BSL performance may be predictable from rotation scores at the outset of the degree, with an advantage for those who already start the SLI program with better MR skills (see, e.g., Kartheiser et al., 2022, who conclude that adult L2 signers can apply pre-existing non-linguistic spatial skills to the sign language they are learning). Regardless of initial MR skills, however, the findings suggest that students who do not improve at MR as they advance in the program do not perform as well as those who did. This may be true not only for BSL comprehension but for production as well. Second-year visuospatial WM was also a significant predictor of SRT scores at the final testing point (Figure 4A). Both MR and visuospatial WM are likely implicated in this task, where increasingly complex grammatical constructions in BSL must be reproduced. Furthermore, the BSL-SRT, like the copy-sign task and nonsense sign repetition tasks which were predictive of sign language performance in previous studies (López Gómez et al., 2007; Stone, 2017), involves phonological encoding and perceptuo-motor skills (see also Martinez and Singleton, 2018, who found that visuospatial short-term memory was predictive of sign learning, concluding that perceptuo-motor processes play a big role in individual sign learning). However, we did not replicate the result seen by Stone (2017), whereby initial performance on the phonological encoding task (MLAT Number Learning) was predictive of early BSL module grades.

In terms of SLI performance, we found that initial auditory WM was a promising indicator of second-year SLI grades (Figure 7B), suggesting it may be a useful assessment to conduct at student intake. While a digit span task was also used by Stone (2017) as a control measure of general cognitive ability, we employ it here as a measure of WM. Using an auditory version of the task has allowed us to explore the effects of different modalities in WM that previous SLI aptitude studies have not. There was also a significant correlation between SLI grades and 3D-MR in the third year (*r*^2^ = 0.54, *t* = 2.85, *p* = 0.029). The third-year BSL-to-English interpreting task was also significantly correlated with second-year 2D-MR (Figure 8A), and the correlation with pre-degree 3D-MR was also very high (*r*^2^ = 0.48, *t* = 2.004, *p* = 0.101; Figure 8D). The relationships here between MR skill and SLI outcomes were beyond what we had predicted: we had hypothesized that rotation would only be implicated directly in BSL tasks. However, it is plausible that rotation skills required during sign language comprehension and production (e.g., for syntactic and topographic uses of signing space) also come into play during measures of SLI itself. Furthermore, interpreting interactions also involve competent navigation of the spatial relations between interlocutors in physical space, where the viewing angle may be a factor. For example, in group scenarios, MR may be invoked to comprehend signing viewed from a non-frontal angle (Watkins et al., 2018). Lastly, performance on the SLI task from English to BSL was significantly correlated with second-year visuospatial WM. It may be that WM in different modalities is implicated in different ways during SLI when working in different directions: for example, visuospatial WM could be particularly important while planning and executing sign language production, as required by this task. Visuospatial WM may be required constantly for production in the visuospatial modality during spoken to signed interpreting, whereas when interpreting in the opposite direction, visuospatial WM is only engaged to attend to the spatial relations in signing space and is not required for the processing of specific signs.

Overall, the predictor assessments with the best and most consistent relationships to BSL and SLI performance were the MR tasks, in particular the 3D-MR task, and visuospatial WM. MR tasks were significant or marginally insignificant predictors of all the BSL/SLI outcome measures in this study: BSL grades, BSL sentence reproduction, SLI grades, and interpreting tasks in both directions, suggesting that MR is an essential skill for SLI educators to pay explicit attention to. Second-year visuospatial WM was a significant predictor of final BSL sentence repetition and strongly correlated with English-to-BSL interpreting performance, which we interpret as WM in the visuospatial modality being necessary for the BSL chunking, planning, and production required during both tasks. Most of the relationships between the cognitive/linguistic assessments and BSL/SLI performance emerged during re-testing at later sessions, although some notable exceptions may point toward skills that have predictive value at the outset of an SLI degree program. Initial 3D-MR skill was strongly correlated with the same two final-year outcomes as second-year visuospatial WM (SRT and English-to-BSL interpreting), highlighting the key role of cognition in the visuospatial modality for tasks involving planning and executing sign language production. We also saw that initial English vocabulary was important early on in L2 BSL learning, as well as a promising relationship between initial auditory WM and second-year SLI grades, suggesting both of these tasks are worth assessing at intake. Although our data are only exploratory, we have some initial evidence that supports Marks (2014) assertion that “[a] case can be made that there are cognitive skills that need to be present upon entry into [SLI] programs and others that can and need to be taught”.

### Implications and future directions

This exploratory study highlights multiple domains worth further attention for SLI educators and researchers. To our knowledge, this is the first longitudinal study of SLI students to take baseline cognitive and linguistic measures before the start of the training program and relate them to performance on sign language and SLI tasks. We saw evidence that MR skill is implicated in not just sign language outcome measures but also in SLI performance, as well as links between visuospatial working memory and sign language production, in particular. We see some evidence that good English skills are initially important for early BSL learning, plus a possible role of initial auditory WM in SLI, which should be investigated by future studies.

Since this is still a preliminary study, however, we do not advocate excluding SLI program applicants at intake based on performance in any of the assessments conducted here. As Robinson (2022) highlights, there are issues with (mostly hearing) SLI educators further restricting the pool of potential SLI students at intake, particularly when interpreter demand already exceeds supply. Nevertheless, initial SLI aptitude testing could help to instead highlight other related careers that do not involve SLI, which may be more appropriate for some candidates, before struggling with a lengthy degree program with its associated expense. Future studies testing (visuospatial) cognitive skills at SLI course intake should also consider the additional stresses of assessments at interviews and issues, such as stereotype threat, i.e., where performance is affected by the awareness of a negative stereotype about one’s social group. For example, women are often perceived to have poorer visuospatial skills, yet Moè and Pazzaglia (2006) found that the gender effect in MR could be negated by explicitly contradicting such stereotypes in task instructions. Such perceptions and stereotypes around visuospatial skills should be a consideration for aptitude testing, given that most (BSL) interpreters are women (Napier et al., 2021), as were most of the SLI students/applicants in this study. Regardless of initial baseline performance, our preliminary results should make SLI training programs aware of skills that would be worth tracking in their students, as well as the possibility to offer the additional targeted practice of skills, that are likely to improve throughout SLI training. Since it is now well-established that MR skill improves in tandem with sign language learning, it is also plausible that we could speed up this process by explicitly including rotation practice on assignments, tasks, or games, whether in a sign language context or not. This could be implicit practice with comprehension of sign language from different viewing angles in group or dialogue situations, where MR is likely implicated (see e.g., Watkins and Thompson, 2019). Alternatively, this could take the form of explicit training using gamified versions of MR tasks, like the ones used here, to try to boost performance, which should, in turn, feedback into signing and interpreting performance (see e.g., Passig and Eden, 2001). Furthermore, SLI educators can use these results to diversify the teaching and learning experience to better support students’ development in these areas.

The title of Stone (2017), “the trials and tribulations of a longitudinal study,” bears repeating, because aptitude studies of SLI students are complex endeavors. No single longitudinal study can address all the design, methodology, and data analysis issues. As Stone pointed out, we must be careful when interpreting the results of SLI aptitude studies, because most of the effect sizes are modest due to both the high levels of attrition and the small initial sample sizes. Even without the impacts of the pandemic and the high drop-out rate in SLI degree programs, studies on the SLI student population in the UK are always likely to be small in scale, due to the population to sample from not being very large (around 60 new degree students per year in total). Despite the small *n* in this exploratory study, we hope that our sample is somewhat representative, having tested most of the students across 2 year-groups from two of the three UK universities where SLI programs are taught in degree form. However, issues of sample size and statistical power will likely continue unless an international, multi-center study is organized. In this study, we had hoped to perform the first institution-level comparison in the UK, but participant recruitment and retention proved particularly difficult. Future large-scale longitudinal studies could also be facilitated by using online testing for many of the assessments, which we discovered worked well for students who had the means to take part remotely at later sessions. The tasks hosted on Pavlovia and GoReact were particularly successful. Online aptitude testing could facilitate access to a larger population of SLI students, however, factors, such as equity of access to technology and space to participate online, should be considered carefully. Given the extra adaptations to SLI and sign language teaching programs that were required due to the pandemic (see e.g., Hornstra, 2021; Katz, 2021), and the increasing use of online teaching methods in L2 sign language learning, even pre-pandemic (Ackerman et al., 2018), we hope this preliminary study demonstrates that online SLI aptitude testing is also feasible.

Further improvements to a future larger study could be gained by testing control groups of students on sign language-only degrees without the SLI components, and/or students on other degree programs; for example, a spoken language interpreting course with a comparable ‘placement’ year abroad. This would allow us to tease apart the respective effects of learning BSL vs. learning BSL *and* SLI within a degree program context, as well as any potential effects of simply completing a university degree or interpreting degree. Furthermore, more explicit attempts could be made to retain the participation of students who decide to withdraw from SLI programs. While we did not attempt to re-test students who had left their SLI course at later time points, continuing to include them as participants in the study would allow researchers to make stronger inferences about aptitude and the factors that can be attributed to changes in cognitive and linguistic skills over time. Since Stone (2017) also discovered several differences in skills between his student cohort and his group of experienced interpreters, another important avenue for future research would be to follow SLI program graduates as they transition to the workplace, to pinpoint how long it takes graduates to perform at the level of experienced interpreters. This could help highlight gaps in SLI training curricula.

## Conclusion

Overall, our exploratory study has revealed various new insights about cognitive and linguistic aptitude for L2 sign acquisition and SLI. Crucially, we have tested a range of assessments before the beginning of an SLI training program and followed both their development over time and their impact on signing and interpreting outcomes. Several of our preliminary results are consistent with previous findings suggesting the importance of both phonological encoding and visuospatial WM in SLI student success. We also tested new domains, such as MR, which, to our knowledge, has not been tracked in SLI students before. In particular, 3D-MR showed the biggest improvement over time and was strongly correlated with a range of BSL and SLI outcome measures, as well as there being some indication that pre-degree skill in this domain may be associated with later signing and interpreting performance. We also argue that visuospatial WM and 3D-MR are particularly important for tasks involving sign language production, with implications of modality for broader theories of cognition and language aptitude. These preliminary results will hopefully inform SLI educators about relevant skills to identify and support during training programs, as well as provide a basis for longer-term studies of SLI aptitude through to professional proficiency.

## Data availability statement

The datasets presented in this study can be found in the Open Science Framework (OSF) repository for this manuscript: https://osf.io/kjctg.

## Ethics statement

This study was reviewed and approved by University of Birmingham Science, Technology, Engineering and Mathematics Ethical Review Committee (ERN_18-1170). The participants provided their written informed consent to participate in this study.

## Author contributions

All authors developed the idea for this study. FW wrote the first draft of the manuscript and collected and analyzed the majority of the data, with data collection assistance from RT and SW. SW and CS facilitated initial data collection sessions and created and coded the final interpreting tasks. RT also coded some data and assisted with the analysis. All authors were responsible for revising the article.

## Footnotes

1 Details of the BSL and interpreting modules at the institutions in this study are at the links below. Heriot-Watt University: https://web.archive.org/web/20220124142725/hw.ac.uk/uk/study/undergraduate/british-sign-language-interpreting-translating-and-applied-language.htm University of Wolverhampton: https://web.archive.org/web/20220311152939/wlv.ac.uk/courses/ba-hons-interpreting-british-sign-languageenglish/

2 Effect sizes could only be calculated for 2D-MR where enough participants completed the task at both of the sessions being compared.
